RETRACTED

# Yiqi-Huoxue Granule (YQHX) Downregulates Prothrombotic Factors by Modulating KLF2 and NF-*κ*B in HUVECs following LPS Stimulation

**DOI:** 10.1155/2019/9425183

**Published:** 2019-02-06

**Authors:** Hong Wu, Xinzhou Wang, Shuibo Gao, Liping Dai, Haibin Tong, Haixia Gao, Zhen Lei, Yongjun Han, Zhentao Wang, Lihua Han, Dake Qi

**Affiliations:** ^1^Laboratory of Cell Imaging, Henan University of Chinese Medicine, Zhengzhou 450002, China; ^2^Institute of Cardiovascular Disease, Henan University of Chinese Medicine, Zhengzhou 450002, China; ^3^School of Pharmacy, Henan University of Chinese Medicine, Zhengzhou 450046, China; ^4^College of Life and Environmental Science, Wenzhou University, Wenzhou 325035, China; ^5^Memorial University of Newfoundland, Division of Biomedical Sciences, Faculty of Medicine, Newfoundland, Canada A1B 3V6

## Abstract

The Yiqi-Huoxue granule (YQHX) is a traditional Chinese medication widely used in the therapy of the traditional Chinese medicine diagnosis “Qi deficiency” or “blood stasis” in China. Both these symptoms are related to inflammation, but the mechanisms of YQHX against inflammation are largely unknown. Thus, our present study investigated the effects of YQHX on regulating inflammatory responses induced by lipopolysaccharides (LPS) in HUVECs. Our data found that YQHX remarkably inhibits the production of prothrombotic factors, plasminogen activator inhibitor-1 (PAI-1) and tissue factor (TF), while it upregulates the protein expression of Kruppel-like factor 2 (KLF2). The increase in PAI-1 and TF was significantly attenuated through a transgenic knockdown in KLF2 with a Lenti-shKLF2 vector. YQHX also decreases the phosphorylation of nuclear factor-*κ*B (NF-*κ*B) p65 and I*κ*B following LPS stimulation, and it effectively suppresses PAI-1 and TF via a NF-*κ*B-dependent mechanism. Taken together, our results suggest that YQHX provides a notable antithrombotic activity via regulating the KLF2 expression and NF-*κ*B signaling pathway in HUVECs. The KLF2 and NF-*κ*B may be potential therapeutic targets for interventions of inflammation associated with atherosclerosis.

## 1. Introduction

Acute ischemic heart disease is a leading cause of death and disability worldwide [1]. It is usually associated with luminal thrombosis resulting from vulnerable atherosclerotic erosion or plaque rupture initiated by endothelial dysfunction [2]. Chronic inflammation is involved in the development of luminal thrombosis [3], due to its role in exacerbating endothelial injury and provoking atherosclerotic plaque rupture [2, 4]. However, current antiatherosclerotic agents and antiplatelet therapy only prevent the physical formation of thrombosis [5, 6], but do not alleviate inflammation or endothelial dysfunction. Thus, developing new strategies aimed at protecting against inflammation and endothelial dysfunction may have important clinical implications in antithrombotic therapies.

RETRACTED

The Yiqi-Huoxue granule (YQHX) is a traditional Chinese medication widely used in the therapy of the traditional Chinese medicine diagnosis “Qi deficiency” or “blood stasis” in China. It is composed of Ginseng Radix et Rhizoma (*Panax ginseng* C. A. Mey), Astragali Radix (*Astragalus membranaceus* (Fisch.) Bge.), Paeoniae Rubra Radix (*Paeonia veitchii* Lynch), and Carthami Flos (*Carthamus tinctorius* L.). The Paeoniae Rubra Radix, Carthami Flos, and Ginseng Radix et Rhizoma extracts have been recognized to produce antithrombotic effects [7–9]. The components of Ginseng Radix et Rhizoma and Astragali Radix in YQHX are effective to inhibit inflammatory responses [10, 11]. Our previous studies have demonstrated that YQHX could inhibit the expression of prothrombotic factors, plasminogen activator inhibitor-1 (PAI-1) and tissue factor (TF), induced by thrombin in human umbilical vein endothelial cells (HUVECs) [12]. It also reduces platelet aggregation associated with myocardial infarction in rats [13]. However, so far, it is largely unknown if the antithrombotic effect of YQHX is associated with its anti-inflammatory activity.

Kruppel-like factor 2 (KLF2) is a transcriptional regulator highly expressed in endothelial cells. Overexpression of KLF2 prolongs thrombotic time and mediates *in vivo* rapamycin-induced arterial thrombosis in mice [14, 15]. Conversely, KLF2 deficiency inhibits antithrombotic genes [16]. KLF2 also mediates acute and chronic inflammations [17, 18]. The anti-inflammatory effects of KLF2 mechanistically are linked to the suppression of nuclear factor-kappa B (NF-*κ*B) signaling [17, 19] that regulates a variety of genes related to inflammatory responses [20, 21]. Thus, KLF2 may be a key thrombotic regulator due to its effects on regulating both endothelial function and inflammation.

Lipopolysaccharide (LPS) is a component of Gram-negativebacteria. It alters the fibrinolytic system leading to a procoagulant state or thrombosis [22, 23]. LPS stimulates both proinflammatory mediators [24, 25] and prothrombotic factors [26, 27]. In the present study, we used a LPS-incubatedendothelial cell model to mimic inflammatory conditions in human atherosclerotic lesions. We investigated the effects of YQHX on regulating the NF-*κ*B signaling pathway and KLF2 expression in response to inflammatory stimulation. We also examined if the production of prothrombotic factors PAI-1 and TF could function as a downstream readout to test the potential therapeutic effects of YQHX against cardiovascular diseases.

RETRACTED

## 2. Materials and Methods

### 2.1. Reagents

Endothelial cell culture media (ECM), endothelial cell growth supplies (ECGS), and fetal bovine serum (FBS) were purchased from ScienCell Research Laboratories (ScienCell, CA, USA) or Gibco (Gibco, CA, USA). All of the chemicals, including LPS, simvastatin (ST), pyrrolidine dithiocarbamate (PDTC), and 3-(4,5-dimethyl-2-thiazolyl)-2, and 5-diphenyl-2-H-tetrazolium bromide (MTT) dye, were purchased from Sigma-Aldrich (St. Louis, MO, USA). The antibodies against PAI-1 (sc-5297), TF (sc-393657), KLF2 (sc-28675), p65 (sc-109), p-p65 (sc-33020), I*κ*B (sc-371), p-I*κ*B (sc-8404), GAPDH (sc-47724), and *β*-actin (sc-47778) were obtained from Santa Cruz Biotechnology (Santa Cruz, CA, USA). Horseradish peroxidase- (HRP-) conjugated anti-mouse IgG (SA00001-1) and anti-rabbit IgG (SA00001-2) antibodies were purchased from Proteintech Biotechnology (Proteintech Ltd., Wuhan, China). Lipofectamine 2000 was obtained from Thermo Fisher Scientific (Thermo, MA, USA). YQHX, composed of Ginseng Radix et Rhizoma, Astragali Radix, Paeoniae Rubra Radix, and Carthami Flos, was produced by Sichuan Neo-Green Pharmaceutical Technology Development Co., Ltd. (Sichuan, China). It was freshly prepared in a phosphate-buffered solution before use.

### 2.2. HUVECs

The HUVECs were purchased from ScienCell Research Laboratories (ScienCell, CA, USA), and they were cultured in an incubator at 37°C with 5% CO_2_ in ECM medium supplemented with 5% FBS and 0.03 mg/ml ECGS. The HUVECs (around 70-80% confluence) were incubated with YQHX (from 0.25 to 1.25 mg/ml) and ST (3 *μ*M) for 3 hours. This was followed by LPS stimulation (25 *μ*g/ml) for 12 hours.

### 2.3. Cell Viability

The HUVECs were seeded in 96-well plates with a density of 0.7 × 10^4^ cells/well and cultured overnight. The cells were then incubated with YQHX at a concentration of 0-10.0 mg/ml prior to treatment with 10 *μ*l of MTT. The absorbance at 570 nm was detected using a microplate reader (Thermo Fisher Scientific, Waltham, USA).

### 2.4. Transfection of HUVECs

293T cells in the logarithmic growth phase were cotransfected with recombinant pBOB plasmid, PAX-2, and VSV-G for 48 h. The supernatant was centrifuged at 4000*g* for 10 min at 4°C to remove cell debris and further concentrated to obtain lentivirus. To overexpress KLF2, the HUVECs were infected with lentivirus containing a KLF2-overexpressing sequence (Lenti-KLF2). As shown in Table 1, the KLF2 short hairpin RNA (Lenti-shKLF2, Cyagen Biosciences Inc., Guangzhou, China) was used to knockdown KLF2 as described previously. The cells were also transfected with a scrambled Lenti-GFP as the negative control. The efficiency of transfection was detected with fluorescence microscopy.

RETRACTED

### 2.5. Western Blot Analysis

The cellular lysates extracted from HUVECs were used to quantify protein expression by Western blot. Briefly, the protein concentration was determined by a BCA protein assay kit, and equal amounts of proteins were loaded into 10% SDS-PAGE gels. Following transfer and blocking with 5% skim milk for 1 h at room temperature, the membranes were then incubated with primary antibodies against KLF2 (1 : 200 dilution), PAI-1 (1 : 500 dilution), TF (1 : 500 dilution), p65 (1 : 500 dilution), p-p65 (1 : 500 dilution), I*κ*B (1 : 500 dilution), p-I*κ*B (1 : 500 dilution), GAPDH (1 : 2000 dilution), or *β*-actin (1 : 2000 dilution) overnight at 4°C. Following incubation with a secondary antibody and ECL, the proteins were visualized using a Bio-Rad Gel Doc XR^+^ Imaging System (Bio-Rad, CA, USA). The intensity of the bands was assessed using ImageJ software (available at http://rsbweb.nih.gov/ij/).

### 2.6. Statistical Analysis

The data were analyzed using either parametric test or nonparametric Mann-Whitney *U* test depending on the pattern of data distribution, and the results are presented as the mean ± SD. A *p* value less than 0.05 was considered statistically significant.

## 3. Results

### 3.1. LPS Upregulates PAI-1 and TF Expression in a Time-Dependent Manner

LPS regulates PAI-1 and TF in both cell and animal models [26, 27]. The present study investigated the effects of LPS on regulating the expressions of prothrombotic factors, PAI-1 and TF, in HUVECs. We observed that following LPS stimulation (25 *μ*g/ml), the protein levels of PAI-1 and TF significantly increased in a time-dependent manner in HUVECs (Figure 1). The parallel enhancement of PAI and TF suggests that LPS treatment significantly induces prothrombotic reactions in HUVECs by upregulating both PAI-1 and TF.

### 3.2. YQHX Inhibits LPS-Induced Expressions of PAI-1 and TF in HUVECs

A low concentration of YQHX (no more than 1.25 mg/ml) incubated with HUVECs did not affect cell survival (Figure 2(a)). Thus, we cotreated the cells with YQHX and LPS in order to identify the protective effects of YQHX on regulating LPS-induced prothrombotic reactions. Our previous study has demonstrated that YQHX could inhibit thrombin-induced PAI-1 and TF expressions in HUVECs [12]. Our present findings further indicate that YQHX at a low concentration can inhibit LPS-induced PAI-1 and TF (Figure 2(b)). The inhibitory effect of YQHX on both prothrombotic factors PAI-1 and TF is similar to the effect of simvastatin (ST), which is an HMG CoA reductase inhibitor [28] (Figure 2(b)).

RETRACTED

### 3.3. YQHX Inhibits LPS-Induced PAI-1 and TF Expression through KLF2

KLF2 regulates both acute and chronic inflammation and owns antithrombotic properties [17, 18]. LPS treatment significantly reduced the expression of KLF2 in HUVECs (Figure 3(a)). In the present study, we then overexpressed KLF2 in HUVECs to identify its effect on the regulation of the prothrombotic factors PAI-1 and TF. Indeed, Lenti-KLF2 transduction in HUVECs upregulates the KLF2 expression in the protein level (Figure 3(b)). It significantly suppresses the expression of PAI-1 and TF with or without LPS stimulation (Figure 3(c)). In contrast, shRNA targeting KLF2 downregulates the expression of KLF2 in HUVECs (Figure 4(a)), which results in increased PAI-1 and TF expression in the presence or absence of LPS (Figure 4(b)).

At the concentration range of 0.25 mg/ml to 1.25 mg/ml, YQHX was able to overcome the attenuation of KLF2 expression caused by LPS (Figure 3(a)), which is associated with the attenuation of PAI-1 and TF expression. The knockdown of KLF2 with Lenti-shKLF2 failed to inhibit PAI-1 and TF, suggesting that YQHX might modulate the expression of prothrombotic factors through the upregulation of KLF2.

### 3.4. YQHX Inhibits the Phosphorylation of NF-*κ*B p65 and I*κ*B

The activation of the NF-*κ*B signaling pathway is initiated by I*κ*B phosphorylation and degradation. To explore if YQHX regulates the prothrombotic factors by the NF-*κ*B signaling pathway, the phosphorylation levels of NF-*κ*B p65 and I*κ*B were quantified by Western blot. Our data suggest that LPS treatment for 3 hours in HUVECs increased the phosphorylation of NF-*κ*B p65 and I*κ*B, and this was significantly inhibited by YQHX at a concentration range of 0.25 to 1.25 mg/ml (Figure 5). The inhibition of phosphorylation of NF-*κ*B p65 and I*κ*B was more robust following a higher concentration (1.25 mg/ml) of YQHX treatment compared to a lower concentration (0.25 mg/ml) (Figure 5). The high concentration of YQHX displayed the same inhibitory effect on the NF-*κ*B signaling pathway as simvastatin, which is a well-known NF-*κ*B-specific inhibitor. Together, our data suggest that YQHX inhibits LPS-induced inflammation by repressing the activation of the NF-*κ*B signaling pathway in a dose-dependent manner.

### 3.5. YQHX Inhibits PAI-1 and TF through an NF-*κ*B-Dependent Mechanism

NF-*κ*B regulates KLF2 expression, and KLF2 inhibits PAI-1 and TF. Therefore, we investigated if YQHX inhibits the LPS-induced expression of PAI-1 and TF through the NF-*κ*B signaling pathway. Inhibition of the NF-*κ*B pathway by PDTC, which is a specific inhibitor of NF-*κ*B, successfully reversed the reduction in KLF2 expression caused by LPS (Figure 6). This suggests that the NF-*κ*B pathway is important in mediating KLF2 expression. Interestingly, the upregulated levels of KLF2 following treatments with PDTC and YQHX were not comparable. The effects of YQHX on KLF2 seem more robust (Figure 6). Furthermore, cotreatment with PDTC and YQHX impeded the ability of YQHX to increase KLF2 expression. This suggests that the upregulation of KLF2 by YQHX is partially mediated by the NF-*κ*B pathway. We also observed that treatment with PDTC significantly reduced the expression of PAI-1 and TF, and PDTC partially attenuates the effects of YQHX on PAI-1 and TF (Figure 6). Together, our results indicate that YQHX may play a key role in modulating the expression of PAI-1 and TF through an NF-*κ*B-dependent mechanism.

RETRACTED

### 3.6. The Schematic Mechanism of YQHX's Antithrombotic Effects following LPS Stimulation

LPS binds with the cell membrane receptor, TLR4, and activates the NF-*κ*B pathway through a MyD88-dependent pathway. NF-*κ*B then binds with p65 to form a complex, which is further translocated into the nucleus to inhibit KLF2 gene transcription. The KLF2 negatively regulates PAI-1 and TF genes. P65 indirectly promotes the expression of PAI-1 and TF. YQHX downregulates LPS-induced prothrombotic factors through an NF-*κ*B/KLF2 pathway (Figure 7).

## 4. Discussion

Chinese herbs have been used to prevent cardiovascular diseases for thousands of years in China. YQHX is exclusively prescribed as a traditional Chinese medication for blood stasis of cardiovascular disease in the clinical practice in China. The present study is the first to demonstrate that YQHX attenuates the expression of prothrombotic factors, PAI-1 and TF, following LPS stimulation. YQHX mediates the NF-*κ*B/KLF2 pathway leading to the reduction of the PAI-1 and TF expression in HUVECs. Our study may provide an important insight into the utilization of traditional Chinese medicine in the prevention of thrombosis formation driven by inflammation.

Increasing evidence suggests that inflammation plays a critical role in plaque stability, which eventually leads to rupture and thrombosis [29, 30]. Increased expression of TF and PAI-1 in the endothelium and circulating inflammatory cells might accelerate thrombosis enlargement in patients with acute coronary syndrome (ACS) [31]. Statins have been recognized to have anti-inflammatory effects independent of their hypolipidemic actions [32]. However, patients with ACS still remain vulnerable even following statin treatment. Ginsenoside Rb1, which is extracted from Ginseng Radix et Rhizoma, was found to potentially inhibit inflammatory responses by skewing macrophages toward the M2 phenotype [33]. The Astragali Radix polysaccharide significantly reduces LPS-induced gene expression of tumor necrosis factor alpha (TNF-*α*) and interleukin-8 [34]. The extracts of Carthami Flos also possess remarkable anti-inflammatory activity [35]. These findings demonstrate that active extracts from Chinese herbs may regulate inflammation. In fact, a traditional Chinese medicine, Xiangqi Tang (XQT), contains the above active components, and it has an anti-inflammatory function in LPS-treated rat cardiac microvascular endothelial cells. It inhibits the secretion of prothrombotic genes, such as TF and PAI-1, and inflammatory factors, such as TNF-*α* and intercellular cell adhesion molecule-1 (ICAM-1) [36]. The previous study also found that Tongqiaohuoxue decoction (THD), which includes Ginseng Radix et Rhizoma, Astragali Radix, Paeoniae Rubra Radix, and Carthami Flos, also exerts anti-inflammatory and antithrombotic effects by regulating PAI-1 and fibrinolysis [37].

RETRACTED

KLF2 functions as a “molecular switch” to regulate vascular homeostasis by maintaining the integrity of the endothelial barrier under physiological and pathological conditions [16]. KLF2 overexpression represses PAI-1 and TF gene expression with or without cytokine TNF-*α* stimulation [16]. Statins and shear stress also provide antithrombotic actions by stimulating the KLF2 expression in a dose-dependent manner [38–40]. Thus, the upregulation of KLF2 may be a potential therapeutic strategy to limit thrombosis. The present study is the first to demonstrate that YQHX has anti-inflammatory and antithrombotic effects through a KLF2-dependent mechanism. Upregulation of the KLF2 expression by YQHX markedly decreased the production of PAI-1 and TF induced by LPS stimulation, and transgenic knockdown of KLF2 reversed the antithrombotic effects of YQHX.

Typically, NF-*κ*B heterodimers are sequestered with the repressive protein I*κ*Bs and are inactive in the cytoplasm. Various inflammatory stimuli activate the NF-*κ*B pathway by inducing the phosphorylation and degradation of I*κ*Bs [41, 42]. The activation of NF-*κ*B facilitates the expressions of proinflammatory genes during chronic inflammation and atherosclerotic development [43]. Thus, the suppression of NF-*κ*B is an important strategy for overcoming inflammation [44–46]. Previous studies have indicated that the Chinese traditional medicine, XQT, and its active components promote anti-inflammatory effects by inhibiting mitogen-activated protein kinase (MAPK) and NF-*κ*B signaling pathways [36]. Our results are the first to suggest that YQHX suppresses LPS-induced phosphorylation of both NF-*κ*B p65 and I*κ*B. More importantly, YQHX partially inhibits the production of PAI-1 and TF through an NF-*κ*B-dependent mechanism.

RETRACTED

KLF2 inhibits the NF-*κ*B pathway by affecting the recruitment of p300/CBP [19]. In contrast, the NF-*κ*B p65 protein incorporates with histone deacetylase 4 to suppress the levels of KLF2. It primarily acts to inhibit the binding of myocyte enhancer factor 2 (MEF2) with the KLF2 promoter [47]. The present study demonstrated that an inhibitor of NF-*κ*B, PDTC, partially inhibits the upregulation of KLF2 induced by YQHX, suggesting that NF-*κ*B is partially involved in YQHX-regulated KLF2 expression.

## 5. Conclusion

In summary, we demonstrated that YQHX provides anti-inflammatory and antithrombotic effects. It markedly decreases expressions of PAI-1 and TF following stimulation, which are associated with an upregulation of KLF2 in HUVECs. YQHX also inhibits the phosphorylation of NF-*κ*B p65 and I*κ*B proteins, which partially regulate the KLF2 expression. The present findings revealed a mechanism for the inhibitory effects of YQHX on thrombosis formation, suggesting that YQHX may be a promising strategy to prevent inflammation-related diseases.

### 5.1. Limitations of Our Present Study

Our present findings about YQHX are only based on *in vitro* cell culture models. Our future studies will focus on exploring the effects of YQHX against inflammation or endothelial dysfunction in *in vivo* animal models.

## Figures and Tables

**Figure 1:** LPS upregulates the protein level of PAI-1 and TF in HUVECs. The cells were treated with 25 *μ*g/ml LPS from 0 to 12 h. The levels of (a) PAI-1 and (b) TF were determined using Western blot. Data are expressed as means ± SD (*n* = 4). ^#^*p* < 0.05 vs. 0 h.

**Figure 2:** YQHX inhibits LPS-induced PAI-1 and TF expression. (a) HUVECs were incubated with a variable concentration of YQHX (0.625, 1.25, 2.5, 5, and 10 mg/ml) for 15 h. The cell viability was determined by MTT. Data are expressed as means ± SD (*n* = 6). ^##^*p* < 0.01 vs. group without YQHX treatment. (b) HUVECs were pretreated with YQHX (0.25 and 1.25 mg/ml) or ST (3 *μ*M) for 3 h prior to LPS treatment (25 *μ*g/ml) for 12 h. Data are expressed as means ± SD (*n* = 4). ^#^*p* < 0.05 vs. control and ^∗^*p* < 0.05 vs. group with 25 *μ*g/ml LPS.

**Figure 3:** YQHX inhibits LPS-induced PAI and TF expression through KLF2. (a) HUVECs were incubated with YQHX (0.25 and 1.25 mg/ml) or ST (3 *μ*M) for 3 h followed with LPS (25 *μ*g/ml) stimulation for 12 h. (b) HUVECs were infected with Lenti-GFP or Lenti-KLF2 for 24 h. (c) HUVECs were preinfected with Lenti-GFP or Lenti-KLF2, followed by LPS (25 *μ*g/ml) stimulation for 12 h. Cell lysates were then prepared, and Western blot analysis was performed to determine the expressions of KLF2, PAI-1, and TF. Data are expressed as means ± SD (*n* = 4). ^#^*p* < 0.05 vs. control and ^∗^*p* < 0.05 vs. group with 25 *μ*g/ml LPS.

RETRACTED

**Figure 4:** YQHX inhibits the PAI-1 and TF expression in a KLF2-dependent manner. (a) HUVECs were infected with Lenti-GFP or Lenti-shKLF2 for 24 h. (b) HUVECs were infected with Lenti-GFP or Lenti-shKLF2. Then, they were incubated with YQHX (1.25 mg/ml) for 3 h prior to 25 *μ*g/ml LPS stimulation for 12 h. Cell lysates were prepared and subjected to Western blot measurements to determine the expression of KLF2, PAI-1, and TF. Data are expressed as means ± SD (*n* = 4). ^#^*p* < 0.05 vs. control, ^∗^*p* < 0.05 vs. group with 25 *μ*g/ml LPS or LPS plus Lenti-GFP, and ^▲^*p* < 0.05 vs. LPS plus YQHX or LPS plus YQHX and Lenti-GFP.

**Figure 5:** YQHX regulates the phosphorylation of NF-*κ*B p65 and I*κ*B. HUVECs were pretreated with YQHX (0.25 and 1.25 mg/ml) or ST (3 *μ*M) for 3 h before being exposed to LPS (25 *μ*g/ml) for 3 h. Cell lysates were prepared and subjected to Western blot analysis to determine the phosphorylation levels of (a) NF-*κ*B p65 and (b) I*κ*B proteins. Data are expressed as means ± SD (*n* = 4). ^#^*p* < 0.05 vs. control and ^∗^*p* < 0.05 vs. group with 25 *μ*g/ml LPS.

**Figure 6:** YQHX inhibits LPS-induced PAI and TF expression through an NF-*κ*B-dependent mechanism. HUVECs were incubated with 1.25 mg/ml of YQHX or 3 *μ*M of PDTC for 3 h prior to the treatment of LPS (25 *μ*g/ml) for 12 h. Cell lysates were prepared and immunoblotted to determine the expression of KLF2, PAI-1, and TF. Data are expressed as means ± SD (*n* = 4). ^#^*p* < 0.05 vs. control and ^∗^*p* < 0.05 vs. group with 25 *μ*g/ml LPS.

**Figure 7:** Schematic mechanisms of YQHX's antithrombotic effects.

**Table 1:** The sequence of specific KLF2 shRNAs used in the present study. All of the shRNAs correspond to *Homo sapiens*.

Name	Sense (5′-3′)	Antisense (5′-3′)
KLF2 (shRNA1)	GCTGCACATGAAACGGCACAT	ATGTGCCGTTTCATGTGCAGC
KLF2 (shRNA2)	TTGTGATGCCTTGTGAGAAAT	ATTTCTCACAAGGCATCACAA
KLF2 (shRNA3)	CCAAACTGTGACTGGTATTTA	TAAATACCAGTCACAGTTTGG
NC (scramble shRNA)	CCTAAGGTTAAGTCGCCCTCG	CGAGGGCGACTTAACCTTAGG

## Data Availability

The datasets used or analyzed during the current study are available from the corresponding author on reasonable request.
